# Sign Language Recognition for Arabic Alphabets Using Transfer Learning Technique

**DOI:** 10.1155/2022/4567989

**Published:** 2022-04-22

**Authors:** Mohammed Zakariah, Yousef Ajmi Alotaibi, Deepika Koundal, Yanhui Guo, Mohammad Mamun Elahi

**Affiliations:** ^1^College of Computer and Information Sciences, King Saud University, Riyadh, Saudi Arabia; ^2^Department of Computer Engineering, College of Computer and Information Sciences, King Saud University, P.O. Box 57168, Riyadh 21574, Saudi Arabia; ^3^Department of Systemics, University of Petroleum & Energy Studies, Dehradun, India; ^4^University of Illinois, Springfield, USA; ^5^Department of Computer Science and Engineering, United International University, Dhaka, Bangladesh

## Abstract

Sign language is essential for deaf and mute people to communicate with normal people and themselves. As ordinary people tend to ignore the importance of sign language, which is the mere source of communication for the deaf and the mute communities. These people are facing significant downfalls in their lives because of these disabilities or impairments leading to unemployment, severe depression, and several other symptoms. One of the services they are using for communication is the sign language interpreters. But hiring these interpreters is very costly, and therefore, a cheap solution is required for resolving this issue. Therefore, a system has been developed that will use the visual hand dataset based on an Arabic Sign Language and interpret this visual data in textual information. The dataset used consists of 54049 images of Arabic sign language alphabets consisting of 1500\ images per class, and each class represents a different meaning by its hand gesture or sign. Various preprocessing and data augmentation techniques have been applied to the images. The experiments have been performed using various pretrained models on the given dataset. Most of them performed pretty normally and in the final stage, the EfficientNetB4 model has been considered the best fit for the case. Considering the complexity of the dataset, models other than EfficientNetB4 do not perform well due to their lightweight architecture. EfficientNetB4 is a heavy-weight architecture that possesses more complexities comparatively. The best model is exposed with a training accuracy of 98 percent and a testing accuracy of 95 percent.

## 1. Introduction

Over 70 million people use sign language worldwide and an automated process for interpreting it might significantly impact communication between those who use it and those who do not. Sign language is a kind of nonverbal communication that includes other bodily organs. In sign language communication, facial expressions, eye, hand, and lip gestures are used to transmit data. Individuals who are deaf or hard of hearing rely heavily on sign language as a form of communication in their daily lives [1].

As per the World Health Organization, hearing impairment affects 5% of the Earth's population. However, this appears to be a minor figure, it indicates that hearing impairment affects over 460 million individuals worldwide; 34 million of whom are youngsters. Moreover, it is predicted that even by 2050, over 900 million individuals will undergo hearing impairment [2], with 1.1 billion youth at risk of deafness due to noise exposure and other difficulties. Untreated hearing loss costs the world 750 billion US dollars [2]. Based on the severity of the deafness, hearing impairment is classified as mild, moderate, severe, or profound. People with severe or profound hearing impairment cannot attend to others and consequently have communication difficulties. This poor communication could significantly influence the deaf person's mental health, including loneliness, solitude, and dissatisfaction. The deaf society communicates using a gesture-based language known as sign language. Deaf individuals use sign language motions to connect. On the other hand, the hearing society does not recognize these gestures, which creates a communication barrier between a deaf and a hearing individual. There are almost 200 sign languages globally, and sign languages, like spoken languages, vary from each other.

Sign language is a subset of communication used as a medium of interaction by the deaf. Unlike other natural languages, it uses significant bodily motions to communicate messages, known as gestures or signs. To communicate a message, hand and finger gestures, head nodding, shoulder gestures, and facial expressions are employed. Therefore, the proposed work would help deaf people to interact between deaf and deaf or deaf and normal persons. When a deaf or hard-of-hearing person tries to express anything, they use gestures to communicate. Each symbol represents a different letter, word, or emotion. A phrase is formed by the combination of signals, much as the string of words includes words in spoken languages. As a result, sign language is a fully formed natural language with grammar and sentence structure.

Humans need verbal communication to carry out social tasks. Consequently, voiceless or silent (D&M) persons were also incapable of conversing vocally with others. Those who communicate through sign language [3] can overcome this issue. The visual modality to express meaning is known as sign language. The message or feel is represented through a manual sign sequence in conjunction, such as nonmanual elements of the communication. Forms of communication vary from one another and are not mutually exhaustive [4]. Sign languages have their own rules and components, respectively, manual and nonmanual [5, 6]. American Sign Language (ASL), British Sign Language (BSL), Brazilian Sign Language (LIBRAS), Japanese Sign Language (JSL), Arabic Sign Language (ArSL), Hindustan Sign Language (ISL), and Bangla Sign Language (BdSL) are some of the sign languages used across the globe [7]. Sign languages are frequently not understood by those who can talk and hear. Written language plays a minor part in establishing communication between D&M societies and the wider public, as much D&M lacks proficiency in spoken language. Again, this technique is hugely sluggish in immediate and emergency face-to-face conversations [8]. According to reports, over 16 million individuals in Bangladesh are deaf, deafened, or have auditory impairments [9]. They adopt sign language, which most people cannot recognize, to describe their emotions. Interaction between D&M personnel and the general public necessitates translating sign language into a language that the general public can identify.

Deep learning remained a class of learning algorithms developed to describe complex structures by combining numerous nonlinear adjustments. The neural networks linked to building deep neural networks are the essential building blocks of deep learning. These methods have enabled significant progress in sound and picture processing, encompassing face identification, computer vision, voice recognition, automated language processing, text categorization (spam identification), and a diversity of other fields like drug diagnosis and genomics. There are several potential uses. First, deep learning enables computational algorithms with several processing layers to acquire a representation of different abstracted dimensions. Deep learning detects unpredictability in large datasets by using the backpropagation technique to express how a system should modify its inner parameters, which have been used to perform a presentation in each level from the symbolization in the preceding layer. Whereas recurrent networks have cast a flashlight on sequential information, such as voice and text, Deep Convolution Network (DCN) has made significant advances in processing video, picture, audio, and speech. Third, deep learning is often carried out using neural network building. The term “deep” mentions the total number of layers in a network; the more layers, the deeper the system. Third, deep learning is extraordinary in terms of precision. Modern tools and tactics have greatly improved deep learning algorithms to the point where they can outperform human performance. This degree of accuracy is made possible by three innovation-enabling influencing factors: The main aim is to develop a sign language recognition system capable enough of translating the most commonly expressed hand gestures used by deaf or dumb people into textual data. To make these disabled people communicable is the prime objective. The contributions are listed as follows: (i) Several data preprocessing techniques have been applied to make the training process faster and less complex to simplify the model training and evaluation process. (ii) Transformation of inconsistent and irregular Arabic datasets has been done into the proper format by various data augmentation techniques. (iii) The proposed work is based on transfer learning using several architectures pretrained on the ImageNet dataset. Those architectures are customized to make them adaptable for the current problem domain. (iv) The experimental work was carried out to test the pretrained models on the unforeseen data. (v) Several Keras pretrained models have been adopted and convolutional neural network architectures are applied for the given case in which the EfficientNetB4 model has outperformed all other models.

The rest of the paper is organized as follows: Section 2 discusses the related work and different techniques applied in this domain.  Section 3 presents the material and methodology of the proposed work. Subsequently, results and discussion have been presented in Sections 4 and 5, respectively. Finally, the paper is concluded with a conclusion in Section 6.

## 2. Related Work

Arabic is the world's 4th most spoken language (Generates a set Consulting Group 2020). Arabic Sign Language (ArSL) seems to be the certified primary language again for talking and listening impaired in Arab countries. The Arab Federation of the Deaf publicly established this in 2001. Even though Arabic is among the world's main languages, ArSL is still in its early stages. The most common problem that ArSL patients face is “diglossia.” Regional dialects are spoken rather than written languages across every country. As a result, various spoken dialects produced varied ArSLs. They are as abundant as Arab states, yet they share several terms and an alphabet. “ArSL is dependent on the alphabet.” Arabic is a sophisticated and pleasant language and one of the Semitic languages vocalized by about 380 million individuals worldwide as their primary official language. Arabs demonstrate plausible semantic and intellectual unity [10].

The authors in this work [11] concentrated on NN's ability to aid with ArSL hand gesture identification. The purpose of the study was to show the use of several types of NN through living person gesture recognition, including stationary and dynamic indicators. First, they demonstrated the practice of Feed Forward Neural Network (FFNN) and RNN in conjunction with its different topologies, completely and moderately reoccurring systems. They then examined their offered structure; the evaluation results revealed that the suggested form with the entire repeated design does have an implementation with a precision rate of 95% for stationary action recognition.

In this study [12], the authors emphasized the automated acknowledgment of the ArSL alphabets using a picture-based method. In particular, several visual features were investigated to construct an accurate ArSL alphabets sensor. One-Versus-All SVM received the extracted visible tags. The results revealed that the Histogram of Oriented Gradients (HOG) signifier outruns other characteristics. As a result, the ArSL gestures system trained by One-Versus-All SVM using HOG identifiers was developed in this study. The authors in this work [13] used the Kinect Sensor to make a Real-Time System for automatic ArSL identification structure based on the Dynamic Time Warping coordination method. The program does not use any power/data gloves. Many trials were used to detect for a lexicon of 30 distinct phrases specifically produced signals again from standardized ArSL. The architecture could function in three means: digitally, signer-independent, and signer-dependent. They used the Dynamic Time Warping coordination method to differentiate between indications. The tests showed that the current version has a high detection score for each option. The framework achieved a detection accuracy of 97.58 percent and a ratio of error of 2.42 percent for signer-dependent. The algorithm then achieved a detection accuracy of 95.25 percent and a ratio of error of 4.75 percent for signer-independent recognition. In some other works conducted by [14, 15], various aspects of human-computer interactions were discussed.

Alternative techniques to sign lingual identification are focused on Hidden Markov Models, like studies from 2011 that identify Arabic Sign Language including the efficiency of up to 82.22 percent [16]. Some other studies that used Hidden Markov Models can be found in [17]. At the same time, in [18], a five-stage procedure for an Arabic sign language translator was published, concentrating on background subtraction of transcription, magnitude, or partially invariant, and achieving an efficiency of 91.3 percent. Almasre and Al-Nuaim employed unique detectors like the Microsoft Kinect or Leap Motion Detectors for record-keeping throughout one's hand-gesturing system to identify 28 Arabic Sign Language motions [19]. Recent work upon Arabic sign language identification has been revealed throughout [20]. Many CNNs have been formed and offered input from an imaging system that contained the elevation and breadth of items and their intensity. The figures are instead processed by a CNN based on the frame rate of the depth footage, which also determines how extensive the system is. Lower frame rates result in less depth, whereas faster refresh rates result in further detail.

In this work [21], a novel model was introduced for Arabic Sign Language Acknowledgment in 2019 utilizing Convolutional Neural Network (CNN) to recognize 28 Arabic letters and numerals ranging from 0 to 10 from an image dataset of 7869 pictures. The suggested framework had seven layers and was instructed numerous times on various training-testing variations, with the highest correctness seeming to be 90.02 percent with a picture training data of 80%. Eventually, the researchers contrasted with other methods, demonstrating the suggested model's benefit. CNN is a deep neural network category that is most widely used in computer field vision. Vision-based techniques primarily concentrate on acquired pictures of the motion and extract the principal characteristic to recognize it. This technology has been used to solve a variety of problems involving superresolution, picture segmentation and semantic breakdown, multimedia systems, and emotion identification [22–24]. In a similar effort [25], Oyedotun and Khashman were among the few well-known scholars that employed CNN in conjunction with Stacked Denoising Autoencoder (SDAE) to recognize 24 hand motions in American Sign Language (ASL) obtained from a communal record. On the other hand, Pigou et al. proposed using Convolutional Neural Network (CNN) to identify Italian sign language [8]. However, Hu et al. had developed a suggestion for the design of hybrid CNN and RNN to preserve the temporal features correctly for the electromyogram signal, which addresses the issue of action identification. Another work [26] describes an extraordinary CNN model that automatically detects numbers relying on hand signals and communicates the specific outcome in the Bangla language, which is followed in this study. In a similar work [27], a CRNN module for hand pose estimation is conducted. There is also a suggestion in [28] to employ transfer learning on data acquired from many individuals, simultaneously utilizing a deep-learning system to understand discriminant traits discovered in massive datasets. A deep convolutional neural network-based Bernoulli heatmap for head pose estimation was conducted by [29]. Another work [30] related to 3D separable convolutional neural network for dynamic hand gesture recognition is used for recognizing the hand gesture. Another work [31] applied flexible strain sensors for wearable hand gesture recognition, which is the latest in this field of research. Further to the latest work-related hand gesture, the authors here [32] have applied deformable convolution neural networks. Fingerprint detection [33] for the recognition of hand gestures is another latest work proposed for HCI. A lightweight neural network [34] is applied for hand gesture recognition. Geometric features learning [35] is another technique to recognize hand gestures. In [36], a consistent identification system is suggested employing the *K*-nearest neighbor classifier and statistical feature extraction approach for the Arabic sign language as another methodology for recognizing the Arabic sign language. Sadly, the fundamental disadvantage of Tubaiz's technique is that consumers are forced to utilize instrumented hand gloves to collect the specific gesture's details, which frequently creates excellent suffering to the consumer. Following that, [37] suggests developing an instrumented glove to create an Arabic sign language recognition system. They presented constant detection of Arabic sign language employing hidden Markov models and spatiotemporal characteristics. Hand pose estimation with a multiscale network was proposed by [38]. Similarly, [39] studied translation from Arabic sign language to text, which may be utilized on portable devices. The automated identification of Arabic sign language utilizing sensor and image techniques is reported in [40]. In [41], using two depth sensors to identify Arabic Sign Language (ArSL) hand movements proposes a flexible Arabic Sign Language identification structure based on two machine learning algorithms that use Microsoft Kinect. Furthermore, the current CNN technique to Arabic sign language has been unparalleled in the sign language study arena [42]. As a result, the objective of this study is to build a vision-based organization that recognizes Arabic hand sign-based letters and converts them into Arabic language using CNN. For each of the 31 letters of Arabic sign language, a collection of 100 photos in the training set and 25 pictures in the test set is constructed. Several hyperparameter combinations evaluate the proposed system to get the best outcomes with the lowest amount of training duration.

## 3. Material and Methods

### 3.1. Dataset

The dataset consists of 54049 images of Arabic sign language alphabets performed by more than 40 people for 32 standard Arabic signs and alphabets. The dataset is available at ArSL2018 [43], launched by Prince Mohammad Bin Fahd University, Al Khobar, Saudi Arabia, to be open to Machine Learning and Deep Learning researchers. The number of images per class differs from one type to another. Each distinct hand gesture indicates some meaningful information. There are around 1500 images per class, and each class represents a different meaning by its hand gesture or sign. Pictorially, the sample image of each class and its label is illustrated in Figure 1.

For some storage schemes, 32 folders are created, and each folder consists of around 1500 images incorporating differently aged people's hand gestures in different environments. The directories containing these folders are treated as training and validation datasets for the model, which will be explained later in this section. Before talking about the model used, it is mandatory to undergo data preprocessing to make the dataset more consistent and compatible with the model as an input. So, how the data preprocessing is done is elaborated in the next section.

### 3.2. Methodology

Before talking about the model used, it is mandatory to undergo data preprocessing to make the dataset more consistent and compatible with the model as an input. So, how the data preprocessing is done is elaborated in the next section.

#### 3.2.1. Data Preprocessing

The data preprocessing involves the transformation applied to the data before feeding it to the model for training/testing. So, what changes are performed on the dataset is described below. As already mentioned, the number of images per class differs. This imbalance meant among the classes may degrade the training performance of the model. Thus, there must be an equal number of images among all classes to avoid this imbalance meant. This imbalance is removed by looping over each class folder to get the filenames of all the images per class. 1000 images are picked randomly from the current class folder during each iteration, and the rest are removed. Resultantly, 32000 images are filtered by summing up 1000 images of all the classes. The images contained in each class have the dimensions of (64 × 64). To keep the computations while training less complex and fast, the images can be rescaled into (32 × 32) following the same dimensionality ratio. Rescaling is represented pictorially in Figure 2.

*(1) Data Augmentation*. The data augmentation technique is widely used to increase the size of the training dataset by generating artificial modified versions of the original images from the training dataset. The technique results in a more diverse and consistent sequence of images, further creating more generalized and skillful deep learning models. The technique helps avoid overfitting and underfitting the model by applying several optional modifications to the training images. In this case, the following augmented changes are performed on the training images through ImageDataGenerator provided by the Keras API [44]. This augmentation technique includes the horizontal shifting of the object to the left or right up to the defined limit, as shown in Figure 3.

This step includes the vertical shifting of the targeted object to up and down up to a certain limit, as shown in Figure 4. This augmentation technique involves the random darkening and brightening the images up to a certain limit, as shown in Figure 5. This augmentation technique randomly removes or adds the pixels into the images for zoom in or zoom out up to the provided limitation, as shown in Figure 6.

All the above-mentioned augmentation techniques are performed by passing parameters with their limitations to the ImageDataGenerator class provided by Keras API. The transformations of the original image can be seen in Figure 7. It includes various augmented images generated from the one original image belonging to class “khaa.” These images are then converted into normalized images, and this normalization process is explained in the next section. The data normalization step performs the normalization process on each image of the dataset. Usually, the pixel values in the image range from 0 to 255. But these values must be rescaled before providing these images to the model as an input. So, the normalization will rescale these pixel values in the range of (0, 1). This rescaling will keep the model easy to learn and train fast, and this is represented in Figure 8.

Considering Figure 8, there is some contrast difference between the two images. The normalized image is more precise and brighter than the original image. So, normalized images are more adaptable and easier for the model to train.

*(2) Data Splitting*. The data used to build the model comes from multiple types of datasets. There are three different purposeful datasets for any computer vision project to analyze, compare, and improve the model's performance. In particular, these three different types of datasets are used in various stages of creating any machine learning model. These three distinct datasets are stated below:

Training dataset on which the model is trained for learning weights or features. Initially, the model is fitted on the training dataset, and in our case specifically, 80 percent of the whole dataset is used for the training dataset, which is approximately 25600 images. Validation dataset the model is fitted on this dataset for the unbiased evaluation of itself during training. It validates the model's performance based on how well the model learns its weights before it is used for real-time testing on the testing dataset. In our scenario of sign language recognition, 20 percent of the dataset is used, which is equivalent to 6400 images. Test dataset after the completion of training and validation phenomena is used to examine the performance of the proposed model and measure its efficiency and accuracy and how well the model is trained. Nine hundred sixty samples are used for the test dataset since there are 30 test images for each sign alphabet. This self-generated test set is created to measure the model's ability to generalize. More importantly, this test set is not collected from the 32000 images.

After the dataset is fully preprocessed, it is fed to the model network in a compatible input fashion for training. But to start the training, it is vital for the reader to understand the workflow, as shown in Figure 9.

Before starting this time-consuming process, it is necessary to ensure the best possible selection of the deep neural network considering the problem domain. Various frameworks can be used in this case, like TensorFlow, Keras, PyTorch, and so on. Each framework has its pros and cons; considering the problem domain, Keras is used. So, to ensure the best possible fit, there are several pretrained models available in the Keras library. Those pretrained models are trained at the ImageNet dataset to provide state-of-the-art results in the domain of image classification. So, here the question arises that what is the ImageNet dataset and what classes the ImageNet dataset constitutes are explained briefly in the next section.

#### 3.2.2. Keras Pretrained Models

ImageNet is an extensive collection of annotated images publicly made available for computer vision research. This large-scale collection of images is a critical resource for analyzing, training, and testing the machine learning algorithms. There are around 14 million images, and 1000 categories or classes in this dataset, and this dataset is also used for large-scale visual recognition challenge competitions. The pretrained models provided by the Keras. Applications' Python package is also complex functional models because these applicable models are trained on the ImageNet dataset. These pretrained models can classify any image that falls into these categories of images.

As mentioned before briefly, Keras applications constitute several pretrained deep learning models available in its repository. The pretrained weights are also available alongside these models. So, these models are further used for custom object detection, image classification, and so on. But considering the domain problem, image classifiers are filtered from these pretrained models and not the object detectors because the case requires performing the image classification. The selection is made considering the hand gesture dataset's complexity and nature. The selected pretrained models with their results are mentioned in Table 1.

In Table 1, it is essential to note that all the models are trained using the ImageNet dataset. Every model has its size, accuracy, and several parameters along with the architecture depth. These models are retrained further on the Arabic hand gesture classification dataset comprising 32 classes. After training, the best possible fit is considered for the case. So, the final selection is made after custom-training these models on the given dataset. So, the custom-training begins in the next section. The training was carried out on a 32 GB NVIDIA Quadro P1000 GPU with a learning rate of 0.001.

#### 3.2.3. Model Compilation

This section includes a detailed analysis of how to perform the complex training process to produce state-of-the-art results. Transfer learning is the only choice to custom train the selected Keras pretrained models. So, what transfer learning is and how to perform it is explained in the below section.

*(1) Transfer Learning*. Transfer learning refers to the situation when the knowledge learned in one task or domain is reused to improve the generalization in another domain. From machine learning's perspective, it can be defined as reusing the saved weights of any pretrained model to improve the accuracy or to custom-train your model. To use the weights of any pretrained model, for example, VGG16, EfficientNet, some modifications have to be made to make the model compatible with training on another dataset. The changes performed on the neural network are elaborated in the next part.

The EfficientNet is a convolutional neural network architecture as shown in Figure 10. That uniformly scales all the depth, width, and resolution dimensions. Generally, the model is made wide, deep, and high resolution. This network is scaled up more efficiently, so, gradually, everything is increased. The network consists of 7 blocks, and each one of these blocks further several subblocks. So, these subblocks additionally contain the layers that are the architecture's main building blocks. What modifications are made in this architecture is explained in the next section.

*(2) Modifications in Pretrained Models*. Three modifications are made to make the model ready to train in the given case. Those modifications are briefly explained below.

- Input layer modification
- The input layer is changed considering the dimensions and size of the input images. In the current case, the images are of the size (64, 64), and the ImageDataGenerator class receives the input shape parameter to automatically prepare the input layer of the model to initialize the training process.
- Output layer modification
- The output layer is modified depending upon the number of classes. The number of neurons is equivalent to the number of classes at the output layer.
- Addition of layers
- Some dense (fully connected) layers are added at the bottom of these ready-made architectures just before the output layer to make the model more effective and suitable for use following the complexity and the format of the dataset.

*(3) Optimizer*. An optimizer is a final argument required to compile the model before training phenomena. There are different variants of optimizer available in the Keras library like SGD (stochastic gradient descent), RMS (root mean square), Adam, and so on. For hand gesture recognition, Adam [45] is used. The “Adam” optimizer is used to reduce the loss calculated after each epoch while training. This optimizer uses the stochastic gradient descent method that is based on the adaptive estimation of first-order and second-order moments. This method is computationally efficient, occupies less memory, is invariant to diagonal rescaling of gradients, and is best suited for the problems that require complex processing in terms of data/parameters.

*(4) Loss Function*. The loss function is the necessary argument used in the model compilation. The loss function calculates the training or/and validation losses after each epoch during the training phenomena. This measurement provides the level of goodness that shows how well the model is being trained. An increase in loss degrades the model performance, and a decrease in loss optimizes the model performance. There are several built-in classes available in the Keras library for calculating the loss during training. The selection depends upon the nature of the dataset. In the case of image classification having more than two classes to predict, the “categorical_crossentropy” class is used. This class computes the cross-entropy loss between the ground truth values and the predicted values resulting from model predictions.

*(5) Training Callbacks*. The callbacks are used to perform specific actions at different stages of the training process. These are useful when a developer wants to save model information during or after the training process. These callbacks can be performed before and after the single batch, start or end of an epoch, and so on. The Keras library provides various callbacks, but in this case, few callbacks are considered to be used during the training of the model. These callbacks have their specific functionality and purpose, briefly explained below.

*(6) Model Checkpoint*. This callback is used to save the Keras model or the model weights after some intervals during the training process. The save model file can be used further to load and start the training again or for testing or evaluation purposes. This callback can be used in several ways, providing the optional arguments to the callback class. The options are described precisely below. Whether to save the model possessing the best performance or to save the model file after each epoch, disregarding the model performance. In the specific case, the best model file is protected if the model is improved as compared to past versions. The callback can only be used based on the monitored quantity. The quantity to be monitored and whether it should be maximized or minimized. The monitored amount can have four options: train_accuracy, train_loss, validation_accuracy, and validation loss. In this case, validation_accuracy is termed as a monitored quantity. The callback also provides the option of at what frequency it should save the model file. The model checkpoint file is saved after each epoch analyzing the validation accuracy. So, there are several other options available to use this callback, but the above-mentioned options are used in the given case.

*(7) Early Stopping*. This callback is used to stop the training process automatically when model performance stops improving up to a specific limit based on some monitored quantity. As previously mentioned, the amount monitored in the given case is validation accuracy. The training process terminates when the validation accuracy stops improving up to a certain number of epochs. Several optional arguments are used to perform this early stopping, and those options are explained. The validation accuracy (monitored quantity) qualifies to be improved when increased with the minimum change. This minimum charge can be passed as a parameter to the early stopping class as a min_delta argument. This min_delta option controls the threshold of change to be qualified as improved validation accuracy. The patience option controls when the training process is terminated automatically. The training automatically ends when the model performance starts degrading for the defined number of epochs. This termination is caused when model degradation crosses the patient value specified in the early stopping class.

*(8) CSV Logger*. This callback is used to save the training statistics in a file at runtime during training phenomena. The result of each epoch is held in that file. In addition, a comma-separated log file is used to save the results after each epoch in the given case. So, the callbacks mentioned above are passed as an array to fit() function to apply these callback operations to hunt the most optimal model better and save the evaluation matrices. After defining the training and validation generators to make the dataset ready to train, finalizing the optimizer, loss function, and applying the training callbacks, the model compiles successfully. After successful compilation, the Keras model is now ready to train, which is explained in the next section.

## 4. Experiments and Discussion

### 4.1. Model Training

At this stage, the model instance is fitted to the fit() function to start the training process. This function trains the model for a fixed number of epochs (iterations on a dataset) using training and validation generators that incorporate the preprocessed images and other required attributes as mentioned in the preceding sections. The model had been trained for 25–30 epochs in almost 10 hours, and each epoch took 2000 steps to complete. The number of steps per epoch depends upon the batch size and the training number of images. For example, the number of training images is 128000, and the batch size is 64. The number of steps per epoch is calculated by dividing the number of training images by batch size, equivalent to 2000 steps in the given case.

### 4.2. Performance Metric for Evaluating the Model

Also, we used other different evaluation metrics as the precision and recall and *F*1-score to evaluate our model concerning each class individually from the 32 Arabic alphabet sign classes as shown in Table 2.

#### 4.2.1. Precision

It is also known as the Positive Predictive Value. Accuracy is defined as the proportion of correct predictions divided by the total number of correct class values projected. Equation (1) is used to calculate precision.

(1) $$\begin{array}{c} \text{Precision}=\frac{\left(\text{True Positive}\right)}{\left(\text{True Positive}+\text{False Positive}\right)}. \end{array}$$

#### 4.2.2. Recall

It is sometimes referred to as vulnerability. Recall is defined as the proportion of correct predictions divided by the number of correct class values. Equation (2) is used to calculate recall.

(2) $$\begin{array}{c} \text{Recall}=\frac{\left(\text{True Positive}\right)}{\left(\text{True Positive}+\text{False Negative}\right)}. \end{array}$$

#### 4.2.3. *F*1-Score

The *F*-score or *F*-measure is another name for the *F*-score. The *F*1-score represents the balance between precision and recall. Only when the precision and recall numbers both are good does the *F*1-score grow high. *F*1-score values array from 0 to 1, with the greater the number, the greater the classification accuracy.

(3) $$\begin{array}{c} F1-\text{score is calculated by Equation,}\\ F1-\text{score}=\frac{\left(2{}^{*}\text{Precision}{}^{*}\text{Recall}\right)}{\left(\text{Precision Recall}\right)}. \end{array}$$

### 4.3. Model Evaluation

After the model is trained, testing is required to measure the model's real performance on unseen data that the model has not encountered yet. The scikit-learn library provides different programmatic approaches to test the performance of the trained model. The statistical evaluation is done using two methods: confusion matrix and classification report. To describe the performance of the classification model on a test dataset, the classification report is represented in Figure 11.

Figure 11 illustrates the representation of the leading classification matrix on a per-class basis. This visual report gives better and deeper intuition about the classifier's behavior, showing the trained model's functional weaknesses in many analytical aspects. Here, the support column shows the count of test images per class; for example, all classes constitute 1000 test images. The total test samples are 32000. *F*1-score is the mean of precision and recall. The ability of the classifier to find all positive instances (correct predictions) is defined by the recall column numerically. All the classes show the true predictions of more than 95 percent in the recall column except five classes. The report shows the testing accuracy to be 95 percent, which is the real predictive result of our classifier. The accuracy of the other results is explained in Table 3.

To find the best-suited model for the given case, several Keras pretrained models are taken into the trial. Eventually, EfficientNetB4 has the best performance in terms of accuracy and loss. To analyze the best-suited model for the given case, it is recommended to plot the graphs for accuracy and loss. So, the graphical approach is used to represent the whole training history of the model with epoch count on the *x*-axis and the accuracy/loss on the *y*-axis. The parameters on the *y*-axis include validation loss, validation accuracy, training loss, and training accuracy. Figures 12 and 13 provide a deep insight into how well the EfficientNetB4 model is trained. It can be seen that the accuracies in Figure 12 and the losses in Figure 13 are converging towards each other steadily up to the 10th epoch. After the 10th epoch, both the accuracies and losses diverge from each other and thus, indicating that the model has learned the weights well. So, the model stops until the 25th epoch to avoid overfitting because the model has known the input features to better classify the unforeseen hand gestures. The behavior can be seen graphically as below.

After having the graphical analysis on the training and the validation performance of the model, the following general step is to test the model on unforeseen data. The random and unexpected evaluation tests the actual intelligence of the trained model about how well the model has learned from the input information. This unpredictable behavior is explained precisely in the next section.

### 4.4. Comparative Analysis

The previous work done with hand gesture recognition is not so generalized and authentic to use in different environments. Also, based on the dataset, previous papers published include the dataset consisting of not more than 20 classes, but in the given case, the dataset contains around 32 classes constituting nearly 160000 images. In most cases, considering the previous work, the dataset is converted into grayscale images and this dataset transformation sometimes degrades the model performance. Secondly, several data augmentation techniques are applied in the given case to make the solution adaptable to different environments. Concerning generalization versus specialization, the model trained in the current issue is more generalized than the models analyzed in past papers. The datasets and approaches explored in the previous work indicate that the solution is not adaptable and generalized. Therefore, the specialization problem is now resolved because the model is trained in a diverse environment. For the applicability considering the given case, the solution is more applicable than the past work. It can be adapted in real-time environments as well. Briefly, the comparative analysis is summarized in Table 4.

As shown in the above Table 4, the proposed method is better than the 2 methods and better than many in terms of classes.

The novelty of the proposed work is listed as follows: The proposed work is hand gesture recognition using the simple and efficient classifier. It includes the process of retraining the pretrained TensorFlow architectures. It includes the absence of the sensor hardware. Most of the approaches used to perform Sign Language Recognition includes wearing hand data gloves for the acquisition of hand gesture data. Instead, the current approach does not include any hardware but the mandatory camera. The proposed method is highly efficient and feasible for real-time applications. This method includes the current system, which becomes more applicable when hand detection is added. Adding hand detection and tracking stage makes this application more adaptable and comprehensive. The proposed system has a low latency of classifying the hand gestures.

## 5. Discussion

The whole workflow is discussed following the steps of data preprocessing and model training and evaluations. Data augmentation has played a vital role in preventing the training models from being overfitted, thus improving the models' overall performance on the unforeseen dataset. For data augmentation on the image's dataset, 5000 augmented images are generated using 1000 original images per class. Considering the number of classes that is 32, 5000 ^∗^ 32 images are generated using 1000 ^∗^ 32 original dataset. Consequently, 160000 augmented images are generated using 32000 original normalized images and, thus, played a vital role in the prevention of degradation of the models. Other than this, the preprocessing techniques and architecture modifications applied are the crucial steps in successful sign language recognition. The results accomplished are marginally better than the past works. Considering the current and the past work as summarized in Table 4, this solution is more generalized and better as it performs even better on the test (unforeseen) dataset. But most of the past papers include the accuracies for the specific case without augmenting the dataset. Secondly, the model trained in the current work is based on images containing three colors' spaces instead of grayscale images to make the training process faster.

On the contrary, most of the past papers include training on grayscale images. Focusing on the problem domain, the grayscale images may not perform better considering the high similarity index between the given dataset classes. Thirdly, the current work can be made applicable in real time if hand detection and tracking are made possible in this case. So, these are the few reasons why the current work is better than most of the work done in the past on Arabic sign language recognition or classification problems or hand gesture recognition simply. Knowingly, several pretrained models are trained in the flow, but the best fit is concluded in the final and next section.

## 6. Conclusions

The study is concluded to be the best in its way for Arabic sign language recognition. Considering the steps of the workflow, the very first step is image acquisition. The image acquisition involved the acquisition of the original image taken from the test(unforeseen) dataset to be preprocessed further in the next step. The preprocessing step involves several substeps. The first substep in the preprocessing part is to rescale the given original image that matches the input shape of the model architecture. The input shape was finalized to be (64 × 64 × 3), where 3 indicates the number of color spaces or the dimensions of the input image. After rescaling the image, it is normalized by limiting the pixel values between the range (0, 1). The normalization is performed on the input image so that model may find it easy to extract features and propagate them in between the layers of the architecture for fast prediction with a low latency rate. After normalization, the model receives the preprocessed input image and tries to predict the meaningful pattern on which the model is trained at. Finally, the model attempts to predict the relevant trained patterns of the input image through classification. The classification is made by considering the best-known hand gesture with the highest probability of it happening at most. That class with the highest change is the final prediction made by the trained model. So far, several pretrained models have been tried on various given datasets. Most of them performed pretty usually, and the EfficientNetB4 is considered the best fit for the case in the final stage. Considering the complexity of the dataset, models other than EfficientNetB4 do not perform well due to their lightweight architecture. EfficientNetB4 is a heavy-weight architecture that possesses more complexities comparatively. However, due to its ability to perform on the extensive dataset consisting of a high number of classes, it is the high performer among other pretrained models. The best model is exposed with a training accuracy of 98 percent and a testing accuracy of 95 percent. These accuracies are represented in Figures 12 and 13 as the model is evaluated at the final stage. As a future recommendation, we would like to combine various techniques to handle single-hand gesture recognition. The multiple techniques could be MobileNet and ResNet50 architectures. Another recommendation would be to apply these techniques to detect the gestures from both hands.

## Figures and Tables

**Figure 1:** Dataset overview.

**Figure 2:** (a) Original image versus (b) rescaled image.

**Figure 3:** Width-shift augmented images.

**Figure 4:** Height-shifted augmented images.

**Figure 5:** Brightness-ranged augmented images.

**Figure 6:** Zoom-range augmented images.

**Figure 7:** . Augmented images generated from the original image.

**Figure 8:** (a) Original image versus (b) normalized image.

**Figure 9:** The overall flow of the work.

**Figure 10:** EfficientNetB4 architecture.

**Figure 11:** Classification report.

**Figure 12:** Accuracy graph.

**Figure 13:** Loss graph.

**Table 1:** Statistics of Keras pretrained models.

Model	Size (MB)	Top-1 acc	Top-5 acc	Parameters	Depth
Xception	88	0.790	0.945	22,910,480	126
VGG16	528	0.713	0.901	138,357,544	23
ResNet50	98	0.749	0.921	25,636,712	—
InceptionV3	92	0.779	0.937	23,851,7841	159
MobileNet	16	0.704	0.895	4,253,864	88
EfficientNet	29	0.810	0.922	19,466,823	—

**Table 2:** Comparative study.

Reference	Method	No. of samples (train/test)	Accuracy
[46]	Deep learning using R-CNN	6300/1570	93
[47]	Semantic segmentation—CNN	43239/10810	88
[48]	Keras pretrained models—CNN	526190/16000	87
Our approach	EfficientNetB4	128000/32000	95

**Table 3:** Evaluations.

Terms	Precision	Recall	*F*1-score
Accuracy	0.956	0.962	0.95
Macro average	0.95	0.95	0.95
Weighted average	0.95	0.95	0.95

**Table 4:** Comparative analysis (current work and previous work).

Current work	Past work
More generalized solution	Specialized solution [49]
31 classes	Less than 20 classes [49]
The model trained on RGB images	The model trained on grayscale images [49]
Applied data augmentation techniques	No data augmentation techniques [50]
It can be applied in real time	In most cases, not applicable in real time [51]

## Data Availability

The dataset used in this study is taken from [43].
